The article "Pharmaceutical Reagent Inventory Strategy Based on Contract Shelf Life and Patient Demand" was retracted in 2023. Reasons: signs of a paper mill; suspected computer-generated content; unreliable results or conclusions; concerns about the data.

# Pharmaceutical Reagent Inventory Strategy Based on Contract Shelf Life and Patient Demand

**DOI:** 10.1155/2022/5046141

**Published:** 2022-04-21

**Authors:** Lingling Li, Zheng Liu, Qingshan Qian, Zhao Zhao, Yuanjun Zhao

**Affiliations:** ^1^Department of Central Laboratory, Children's Hospital of Shanghai Jiao Tong University, Shanghai, China; ^2^School of Management, Shanghai University of Engineering Science, Shanghai 201620, China; ^3^Odette School of Business, University of Windsor, N9B 3P4, Windsor, Canada; ^4^School of Accounting, Nanjing Audit University, Nanjing 211815, China; ^5^Institute of Intelligent Management Accounting and Internal Control, Nanjing Audit University, Nanjing 211815, China

## Abstract

As the function and R&D level of in vitro diagnostic reagents continue to improve, the need for hospitals for in vitro diagnostic reagents in clinical diagnosis also keeps increasing. However, under the influence of management, process, technology, equipment, materials, employees, and other unexpected disturbing factors, the output of reagents often has random uncertainty, and it is difficult to provide the finished products required by orders on time, in quality and quantity. A secondary supply chain consisting of reagent manufacturers, distributors, and hospitals is constructed, and the inventory control models of in vitro diagnostic reagent supply chain under three strategies of centralized decision-making, hospital-owned inventory, and reagent distributor-managed inventory are established, respectively, and the maximum expected returns of the supply chain system under different strategies are analyzed to achieve the optimal production decision of reagent manufacturers and the optimal procurement decision of hospitals. The results show that reducing the random output probability and patient demand uncertainty has a significant effect on improving the expected return of in vitro diagnostic reagent supply chain, and as the random output probability of reagent manufacturers and patient consumption demand uncertainty increase, the strategy of managing inventory by distributors in collaboration is always better than the strategy of managing inventory by hospitals' own warehouses, which can achieve higher expected return and better inventory quantity, but when the out-of-stock cost of hospitals is too high above a certain threshold, the hospital will tend to adopt the self-inventory strategy.

## 1. Introduction

In vitro diagnostic reagents refer to reagents, kits, calibrators, and quality control products used for in vitro testing of human samples (various body fluids, cells, tissue samples, etc.) in the process of disease prevention, diagnosis, treatment monitoring, prognosis observation, health status evaluation, and prediction of genetic diseases [1]. For the management of in vitro diagnostic reagents, the most ideal state is to ensure that the actual quality is qualified and that there is no backlog, no unstocking, and no expiration in storage. However, in the actual work, in vitro diagnostic reagents, as a special medical supplies, are affected by multiple uncertain factors such as environment, season, and patient demand, and there are unpredictable fluctuations in the usage, while reagent manufacturers are prone to random output risks due to uncertain factors such as technology and personnel, making hospitals experience backlog or out-of-stock phenomenon, or reagent failure due to storage environment not meeting requirements, which makes the normal operation of hospitals adversely affected and the emergency procurement cost of in vitro diagnostic reagents is invariably greatly increased. Therefore, it is of great practical significance to study how to optimize the inventory quantity of in vitro diagnostic reagent supply chain members, achieve the optimal production decision of reagent manufacturers and the optimal procurement decision of hospitals, improve the efficiency of reagent use by patients, and accelerate the inventory turnover of reagents and maximize the overall expected benefits of the supply chain.

The article "Pharmaceutical Reagent Inventory Strategy Based on Contract Shelf Life and Patient Demand" was retracted in 2023. Reasons: signs of a paper mill; suspected computer-generated content; unreliable results or conclusions; concerns about the data.

The issue of supply chain inventory optimization has long been a key academic concern, but most of the existing literature has been studied from the perspective of market demand uncertainty. Lucker and others [2] considered the use of inventory and reserve capacity strategies to manage disruption risk in pharmaceutical supply chains under stochastic demand and pointed out that the optimal risk mitigation strategy depends on product characteristics and supply chain characteristics. Liu [3] discussed the evolutionary game strategy between government and household medical devices in an uncertain demand environment. Kaya [4] also studied the optimal pricing and inventory replenishment strategy of perishable product inventory system under the certainty that demand depends on time and price. Lin et al. [5] compared three different inventory replenishment strategies, namely forecast forward replenishment, reorder point, and material requirement planning, with practical cases. Minoux et al. [6] introduced and studied a general class of multistage optimization problems related to production/inventory management under the Markov uncertainty, showing how to construct state-space representable uncertainty sets at any probability level. Rau et al. [7] proposed a multi-objective green cycle inventory routing model and discussed the impact of inventory management and transportation on environmental costs. Song et al. [8] considered three inventory strategies: push, pull, and “reservation + one time,” and studied how to realize the inventory optimization of risk-averse suppliers and overconfident manufacturers. Xu [9] discussed the optimization strategy of multilevel inventory of fresh agricultural products. Zhao et al. [10] established an inventory control simulation model for a mixed supply chain of process industries represented by metallurgy, petrochemicals, and pharmaceuticals. In addition, many scholars extended intelligent algorithms to the inventory strategy problem, and Liu et al. [11] studied the inventory and path optimization problem of fresh cold chain in the context of energy-saving and emission reduction with the help of genetic algorithm and hybrid algorithm. Shaikh et al. [12] studied a fuzzy inventory model with allowable delayed payments considering inventory backlog and out-of-stock problem with the help of particle swarm algorithm. Hajek et al. [13] constructed a maximized inventory backorder prediction system based on a machine learning model to improve the robustness of storage/inventory cost and sale profit variation. Simic et al. [14] also proposed a particle swarm optimization and purely adaptive search global optimization algorithm for production inventory system model to minimize inventory quantity, value, and production cost. Srivastav et al. [15] used a multi-objective cuckoo search algorithm to optimize the inventory problem for customer order crossover. Zhou [16] used the genetic algorithm to propose that a joint replenishment strategy can be applied to reduce the total cost in multiproduct multilevel inventory.

The article "Pharmaceutical Reagent Inventory Strategy Based on Contract Shelf Life and Patient Demand" was retracted in 2023. Reasons: signs of a paper mill; suspected computer-generated content; unreliable results or conclusions; concerns about the data.

On the other hand, more and more scholars consider the risk of output uncertainty. Ji et al. [17] develop a multidimensional optimization model for parts ordering decision by portraying the optimal ordering quantity under deterministic demand for two types of supply risks: uncertain capacity and stochastic output rate. Asghar et al. [18] develop a stochastic production inventory strategy to achieve the optimization objectives of production quantity, productivity, and manufacturing reliability under variable energy consumption costs. Hilger et al. [19] considered the use of a mixed-integer linear model to optimize stochastic dynamic multiproduct mass production decisions for remanufacturing firms under dynamic production of capacity. Ye et al. [20] analyzed the selection strategies of farmers' optimal decisions in the face of bank credit, trade credit, and portfolio credit by considering farmers' bankruptcy risk and output stochasticity and constructed a decision model of order agriculture supply chain consisting of a single firm and a single farmer with financial constraints. Sun et al. [21] discussed how to solve the new product presale robust pricing problem to cope with volatility risk in an environment of output uncertainty. Nadal-Roig et al. [22] focused on the production decision of pig production enterprises and used a two-stage stochastic programming model to study how to increase the flexibility and coordination of pig production and identify inefficiencies or bottlenecks in the system. Hu et al. [23] developed a multistage stochastic programming model and obtained the optimal stochastic production sequence and resource allocation decision by solving it. Prilutskii et al. [24] constructed a mathematical model framework to study the optimal control problem of a certain type of production system under uncertainty.

The article "Pharmaceutical Reagent Inventory Strategy Based on Contract Shelf Life and Patient Demand" was retracted in 2023. Reasons: signs of a paper mill; suspected computer-generated content; unreliable results or conclusions; concerns about the data.

A synthesis of the above literature reveals that most of the existing studies on supply chain inventory only consider the unilateral effects of output or demand uncertainty and do not address inventory optimization in this specific area of the in vitro diagnostic reagent supply chain. Therefore, to be closer to the operation practice of in vitro diagnostic reagent supply chain, and considering the random output risk of reagent manufacturers and the uncertainty of patients' demand, this study integrates the idea of supplier-managed inventory, and the local distributors of reagent manufacturers manage inventory in cooperation with hospitals, establishes the production decision model of reagent manufacturers and the procurement decision model of hospitals, and conducts comparative analysis with the two inventory management strategies of centralized decision and hospital self-management to improve the overall revenue of in vitro diagnostic reagent supply chain and obtain the optimal production and procurement decision of hospital inventory.

## 2. Scenario Description and Parameter Assumptions

Consider building a secondary supply chain consisting of in vitro diagnostic reagent manufacturers, hospitals, and reagent distributors. Reagent manufacturers are responsible for the production and supply of certain types of in vitro diagnostic reagents to meet the uncertain demand of hospital patients for such reagents, and hospitals can choose two ordering and distribution methods, ordering from reagent manufacturers and being supplied directly by them or ordering from reagent manufacturers and being supplied by their local distributors, as shown in Figure 1. Suppose the hospital submits purchase order *q*_*t*_ to the reagent manufacturer in this demand cycle *t* to meet the demand in the next cycle *t*+1. When the remaining number of reagents in stock of the reagent manufacturer cannot meet the hospital's purchase demand, i e., *q*_*t*_ > *I*_*t*+1_^*h*^, the reagent manufacturer needs to make production decision to determine the output quantity *p*_*t*_ of reagents in the next cycle and register the produced in vitro diagnostic reagents into the inventory (the age of the inventory is calculated from the *t*+1 cycle). Due to uncertainties such as delayed supply of raw materials and enterprise production capacity constraints, this type of in vitro diagnostic reagents may be unqualified or delayed delivery situation, let the random output rate be *η* and *η* ∈ [*a*, *b*], its cumulative distribution function and probability density function are *G*(*η*) and *g*(*η*), respectively, and the mean value is *μ*_*η*_, and then, the effective output quantity of this type of reagents is *ηp*_*t*_. The reagent manufacturer updates the inventory status at the beginning of *t*+1 cycle, ships the reagents according to the hospital purchase order in the previous cycle on a first-in-first-out basis, and calculates the remaining reagent inventory, out-of-stock quantity, and scrap quantity in the production cycle; the hospital receives the products issued by the reagent manufacturer for clinical treatment and diagnosis of patients according to the same FIFO principle and calculates the remaining reagent inventory, out-of-stock quantity, and scrap quantity in the cycle. After that, the hospital issues purchase order and enters the next cycle of purchase, production, and consumption. Drawing on the literature [25–27], it is assumed that patients have random demand for this kind of in vitro diagnostic reagent, and its cumulative distribution and probability density function are *F*(*x*) and *f*(*x*), respectively, with the mean value of *μ*_*ε*_. *I*_*t*+1_^*h*^, *I*_*t*+1_^*d*^, and *I*_*t*+1_^*e*^ are the initial reagent inventory of reagent manufacturers, reagent distributors, and hospitals in cycle *t*+1, respectively, and *I*_*t*+1_ is the overall inventory of in vitro diagnostic reagent supply chain. *w*_*h*_ is the unit wholesale price of reagent manufacturers to hospitals and reagent distributors, *w*_*e*_ is the unit sale price of hospitals, and *c* is the unit production cost of reagent manufacturers; when the reagent manufacturer fails to meet the purchase needs of the hospital and the hospital fails to meet the needs of patients, it will be punished accordingly. *v*_*h*_ and *v*_*e*_ are the unit shortage cost of the reagent manufacturer and the hospital, respectively, and *k* is the unit reagent scrap cost caused by transportation, storage, and other reasons [28–31].

The article "Pharmaceutical Reagent Inventory Strategy Based on Contract Shelf Life and Patient Demand" was retracted in 2023. Reasons: signs of a paper mill; suspected computer-generated content; unreliable results or conclusions; concerns about the data.

## 3. Model Construction and Analysis

### 3.1. Inventory Management Strategy under Centralized Decision-Making

Under centralized decision-making, it is assumed that hospitals and reagent manufacturers are the same management decision-maker to determine the output volume *q*_*t*_^*c*^ and hospital purchase volume *q*_*t*_^*c*^ of such in vitro diagnostic reagents at the same time; i e., the overall total revenue of reagent manufacturers and hospitals is the optimal target, at which time the total revenue ∏^*c*^ of the in vitro diagnostic reagent supply chain is expressed as follows:

(1) $$\begin{array}{c} \prod^{c}=w_{e}\min\left[\varepsilon ,I_{t+1}^{e}+\min\left(q_{t}^{c},I_{t+1}^{h}+\eta p_{t}^{c}\right)\right]-v_{e}{\left[\varepsilon -I_{t+1}^{e}-\min\left(q_{t}^{c},I_{t+1}^{h}+\eta p_{t}^{c}\right)\right]}^{+}\\ -k{\left(I_{t+1}^{h}+\eta p_{t}^{c}-q_{t}^{c}\right)}^{+}-k{\left(I_{t+1}^{e}-\varepsilon \right)}^{+}-cp_{t}^{c}. \end{array}$$

In which, the first term represents the total revenue of the hospital from the sale of the reagent, the second term is the total cost of out-of-stock for the hospital, the third and fourth terms are the total cost of scrap for the reagent manufacturer and the hospital, respectively, and the last term is the total cost of production of the reagent.

**Proposition 1 .**

The expected revenue function *E*(∏^*c*^) of the in vitro diagnostic reagent supply chain under centralized decision-making is a joint concave function about the vendor output volume *p*_*t*_^*c*^ and the hospital purchase volume *q*_*t*_^*c*^. The maximum expected revenue of the in vitro diagnostic reagent supply chain exists when (*p*_*t*_^*c∗*^, *q*_*t*_^*c∗*^) satisfies the following conditions:

(2) $$\begin{array}{c} \left(w_{e}+v_{e}-k\right)\int_{a}^{\left(q_{t}^{c}-I_{t+1}^{h}/p_{t}^{c}\right)}\bar{F}\left(I_{t+1}+\eta p_{t}^{c}\right)\eta g\left(\eta \right)\text{d}\eta =k\int_{\left(q_{t}^{c}-I_{t+1}^{h}/p_{t}^{c}\right)}^{b}\eta g\left(\eta \right)\text{d}\eta +c,\\ \left(w_{e}+v_{e}-k\right)\int_{\left(q_{t}^{c}-I_{t+1}^{h}/p_{t}\right)}^{b}\bar{F}\left(I_{t+1}^{e}+q_{t}^{c}\right)g\left(\eta \right)\text{d}\eta =\bar{G}\left(\frac{q_{t}^{c}-I_{t+1}^{h}}{q_{t}^{c}}\right). \end{array}$$

**Proof**

The expected revenue function of the in vitro diagnostic reagent supply chain under centralized decision-making is transformed by equation (1) as follows:

(3) $$\begin{array}{c} E\left(\prod^{c}\right)=\left(w_{e}+v_{e}-k\right)\left[\int_{a}^{\left(q_{t}^{c}-I_{t+1}^{h}/p_{t}^{c}\right)}\int_{I_{t+1}+\eta p_{t}^{c}}^{+\infty }\left(I_{t+1}+\eta p_{{}_{t}}^{c}-x\right)f\left(x\right)\text{d}xg\left(\eta \right)\text{d}\eta +\int_{\left(q_{t}^{c}-I_{t+1}^{h}/p_{t}^{c}\right)}^{b}\int_{I_{t+1}^{e}+\eta p_{t}^{c}}^{+\infty }\left(I_{t+1}^{e}+q_{t}^{c}-x\right)f\left(x\right)\text{d}xg\left(\eta \right)\text{d}\eta \right]\\ +\mu_{\varepsilon }\left(w_{e}-k\right)-k\int_{\left(q_{t}^{c}-I_{t+1}^{h}/p_{t}\right)}^{b}\left(I_{t+1}^{h}+\eta p_{t}^{c}-q_{t}^{c}\right)g\left(\eta \right)\text{d}\eta -cp_{t}^{c}. \end{array}$$

The partial derivatives of *E*(∏^*c*^) with respect to *p*_*t*_^*c*^ and *q*_*t*_^*c*^ are as follows:

(4) $$\begin{array}{c} \frac{\partial E\left(\prod^{c}\right)}{\partial p_{t}^{c}}=\left(w_{e}+v_{e}-k\right)\int_{a}^{\left(q_{t}^{c}-I_{t+1}^{h}/p_{t}^{c}\right)}\bar{F}\left(I_{t+1}+\eta p_{t}^{c}\right)\eta g\left(\eta \right)\text{d}\eta -k\int_{\left(q_{t}^{c}-I_{t+1}^{h}/p_{t}^{c}\right)}^{b}\eta g\left(\eta \right)\text{d}\eta -c,\\ \frac{\partial E\left(\prod^{c}\right)}{\partial q_{t}^{c}}=\left(w_{e}+v_{e}-k\right)\int_{\left(q_{t}^{c}-I_{t+1}^{h}/p_{t}\right)}^{b}\bar{F}\left(I_{t+1}^{e}+q_{t}^{c}\right)g\left(\eta \right)\text{d}\eta -\bar{G}\left(\frac{q_{t}^{c}-I_{t+1}^{h}}{q_{t}^{c}}\right),\\ A=\frac{\partial^{2}E\left(\prod^{c}\right)}{\partial {\left(p_{t}^{c}\right)}^{2}}\\ =-\left(w_{e}+v_{e}-k\right)\left[\frac{{\left(q_{t}^{c}-I_{t+1}^{h}\right)}^{2}}{{\left(p_{t}^{c}\right)}^{3}}g\left(\frac{q_{t}^{c}-I_{t+1}^{h}}{p_{t}^{c}}\right)\bar{F}\left(I_{t+1}^{e}+q_{t}^{c}\right)+\int_{a}^{q_{t}^{c}-I_{t+1}^{h}/p_{t}^{c}}\eta^{2}f\left(I_{t+1}^{h}+I_{t+1}^{e}+\beta q_{t}^{c}\right)\text{d}\eta \right]\\ -k\frac{{\left(q_{t}^{c}-I_{t+1}^{h}\right)}^{2}}{{\left(p_{t}^{c}\right)}^{3}}g\left(\frac{q_{t}^{c}-I_{t+1}^{h}}{p_{t}^{c}}\right),\\ B=\frac{\partial^{2}E\left(\prod^{c}\right)}{\partial {\left(q_{t}^{c}\right)}^{2}}\\ =-\left(w_{e}+v_{e}-k\right)\left[\frac{\bar{F}\left(I_{t+1}^{e}+q_{t}^{c}\right)}{p_{t}^{c}}g\left(\frac{q_{t}^{c}-I_{t+1}^{h}}{p_{t}^{c}}\right)+f\left(I_{t+1}^{h}+q_{t}^{c}\right)\bar{G}\left(\frac{q_{t}^{c}-I_{t+1}^{h}}{p_{t}^{c}}\right)\right]-kf\left(\frac{q_{t}^{c}-I_{t+1}^{h}}{p_{t}^{c}}\right),\\ C=\frac{\partial^{2}E\left(\prod^{c}\right)}{\partial p_{t}^{c}\partial q_{t}^{c}}\\ =-\left(w_{e}+v_{e}-k\right)\left[\frac{q_{t}^{c}-I_{t+1}^{h}}{{\left(p_{t}^{c}\right)}^{2}}g\left(\frac{q_{t}^{c}-I_{t+1}^{h}}{p_{t}^{c}}\right)\bar{F}\left(I_{t+1}^{e}+q_{{}_{t}}^{c}\right)+k\frac{q_{t}^{c}-I_{t+1}^{h}}{{\left(p_{t}^{c}\right)}^{2}}g\left(\frac{q_{t}^{c}-I_{t+1}^{h}}{p_{t}^{c}}\right)\right]. \end{array}$$

From the assumptions *w*_*e*_+*v*_*e*_ > *k*, when *q*_*t*_^*c*^ > *I*_*t*+1_^*h*^, such that *A* < 0, *B* < 0, *C* > 0, and *AB* − *C*^2^ > 0, that is, from the negative definite of the Hessian matrix, the expected revenue function *E*(∏^*c*^) is a joint concave function about the output volume *p*_*t*_^*c*^ of the reagent manufacturer and the hospital purchase quantity *q*_*t*_^*c*^. When the first-order partial derivative is zero, the optimal solution (*p*_*t*_^*c∗*^, *q*_*t*_^*c∗*^) is obtained.  Proposition 1 shows that there is an optimal solution to maximize the expected return of in vitro diagnostic reagent supply chain under centralized decision-making.

The article "Pharmaceutical Reagent Inventory Strategy Based on Contract Shelf Life and Patient Demand" was retracted in 2023. Reasons: signs of a paper mill; suspected computer-generated content; unreliable results or conclusions; concerns about the data.

### 3.2. Hospital Self-Operated Inventory Strategy

Assuming that the hospital establishes its own warehouse in this situation, the in vitro diagnostic reagents from the manufacturer will be used for patient treatment according to the FIFO storage principle. Consider a Stackelberg game between a hospital and a reagent manufacturer under the condition of perfect information, in which the hospital as the dominant player determines the purchase quantity *q*_*t*_^*e*^ of such in vitro diagnostic reagents, and the manufacturer as the follower determines the output quantity *p*_*t*_^*e*^ according to the hospital's purchase order. The hospital's revenue ∏_*h*_^*e*^ is expressed as follows:

(5) $$\begin{array}{c} \prod_{e}^{e}=w_{e}\min\left[\varepsilon ,I_{t+1}^{e}+\min\left(q_{t}^{e},I_{t+1}^{h}+\eta p_{t}^{e}\right)\right]-w_{h}\min\left(q_{t}^{e},I_{t+1}^{h}+\eta p_{t}^{e}\right)-v_{e}{\left[\varepsilon -I_{t+1}^{e}-\min\left(q_{t}^{e},I_{t+1}^{h}+\eta p_{t}^{e}\right)\right]}^{+}\\ -k{\left[\min\left(q_{t}^{e},I_{t+1}^{h}+\eta p_{t}^{e}\right)+I_{t+1}^{e}-\varepsilon \right]}^{+}+v_{h}{\left(q_{t}^{e}-I_{t+1}^{h}-\eta p_{t}^{e}\right)}^{+}. \end{array}$$

The reagent manufacturer's revenue expressions are as follows:

(6) $$\begin{array}{c} \prod_{\text{h}}^{e}=w_{h}\min\left(q_{t}^{e},I_{t+1}^{h}+\eta p_{t}^{e}\right)-k{\left(I_{t+1}^{h}+\eta p_{t}^{e}-q_{t}^{e}\right)}^{+}-v_{h}{\left(q_{t}^{e}-I_{t+1}^{h}-\eta p_{t}^{e}\right)}^{+}-cp_{t}^{e}. \end{array}$$

That is, the total revenue of the in vitro diagnostic reagent supply chain is as follows:

(7) $$\begin{array}{c} \prod^{e}=\prod_{e}^{e}+\prod_{h}^{e}. \end{array}$$

The reverse induction method to solve the appeal model is used, the production decision of the reagent manufacturer is first analyzed, and then the hospital's order purchasing decision is discussed.

**Proposition 2 .**

Under the hospital-owned inventory strategy, the expected revenue $E\left(\prod_{\bar{h}}^{e}\right)$ of the reagent manufacturer is a concave function with respect to the output quantity *p*_*t*_^*e*^, and there exists a unique optimal solution *p*_*t*_^*e∗*^ such that the expected revenue of the reagent manufacturer is maximized, and the optimal output quantity *p*_*t*_^*e∗*^ satisfies the following conditions.

(8) $$\begin{array}{c} \left(w_{h}+v_{h}\right)\int_{a}^{\left(q_{t}^{e}-I_{t+1}^{h}/p_{t}^{e}\right)}\eta g\left(\eta \right)\text{d}\eta =k\int_{\left(q_{t}^{e}-I_{t+1}^{h}/p_{t}^{e}\right)}^{b}\eta g\left(\eta \right)\text{d}\eta +c. \end{array}$$

**Proof**

The expected revenue function of the reagent manufacturer is given by equation (5):

(9) $$\begin{array}{c} E\left(\prod_{h}^{e}\right)=w_{h}\left[\int_{a}^{\left(q_{t}^{e}-I_{t+1}^{h}/p_{t}^{e}\right)}\left(I_{t+1}^{h}+\eta p_{t}^{c}\right)g\left(\eta \right)\text{d}\eta +\int_{\left(q_{t}^{e}-I_{t+1}^{h}/p_{t}^{e}\right)}^{b}q_{t}^{e}g\left(\eta \right)\text{d}\eta \right]-v_{h}\int_{a}^{\left(q_{t}^{e}-I_{t+1}^{h}/p_{t}^{e}\right)}\left(q_{t}^{e}-I_{t+1}^{h}-\eta p_{t}^{c}\right)g\left(\eta \right)\text{d}\eta \\ -k\int_{\left(q_{t}^{e}-I_{t+1}^{h}/p_{t}^{e}\right)}^{b}\left(I_{t+1}^{h}+\eta p_{t}^{e}-q_{t}^{e}\right)g\left(\eta \right)\text{d}\eta -cp_{t}^{e}. \end{array}$$

The partial derivative of the above formula with respect to *p*_*t*_^*e*^ is as follows:

(10) $$\begin{array}{c} \frac{\partial E\left(\prod_{h}^{e}\right)}{\partial p_{t}^{e}}=\left(w_{h}+v_{h}\right)\int_{a}^{\left(q_{t}^{e}-I_{t+1}^{h}/p_{t}^{e}\right)}\eta g\left(\eta \right)\text{d}\eta -k\int_{\left(q_{t}^{e}-I_{t+1}^{h}/p_{t}^{e}\right)}^{b}\eta g\left(\eta \right)\text{d}\eta -c,\\ \frac{\partial E\left(\prod_{h}^{e}\right)}{\partial p_{t}^{e}}=-\left(w_{h}+v_{h}+k\right)\frac{{\left(q_{t}^{e}-I_{t+1}^{h}\right)}^{3}}{{\left(p_{t}^{e}\right)}^{2}}g\left(\frac{q_{t}^{e}-I_{t+1}^{h}}{p_{t}^{e}}\right)<0. \end{array}$$

It follows that the expected return *E*(∏_*h*_^*e*^) of the reagent manufacturer is a concave function of the output quantity *p*_*t*_^*e*^, and (∂*E*(∏_*h*_^*e*^)/∂*p*_*t*_^*c*^) is monotonically decreasing with respect to *p*_*t*_^*e∗*^ on the interval (0, +*∞*). Since $\underset{p_{t}^{c}⟶0}{\lim}\left(\partial E\left(\prod_{h}^{e}\right)/\partial p_{t}^{c}\right)>0$ and $\underset{p_{t}^{c}⟶\infty }{\lim}\left(\partial E\left(\prod_{h}^{e}\right)/\partial p_{t}^{c}\right)<0$, there exists only one value *p*_*t*_^*e∗*^ on (0, +*∞*) that satisfies the first-order partial derivative equal to zero; i e., there is: (*w*_*h*_+*v*_*h*_)∫_*a*_^(*q*_*t*_^*e*^ − *I*_*t*+1_^*h*^/*p*_*t*_^*e*^)^*ηg*(*η*)d*η* − *k*∫_(*q*_*t*_^*e*^ − *I*_*t*+1_^*h*^/*p*_*t*_^*e*^)_^*b*^*ηg*(*η*)d*η* − *c*=0. It can be seen that reagent manufacturers determine the output volume of such in vitro diagnostic reagents based on the initial inventory, wholesale price, production cost, out-of-stock cost, end-of-life cost, and hospital orders to maximize the expected revenue. According to Proposition 2, the optimal output *p*_*t*_^*e∗*^ increases with the increase in parameters *w*_*h*_, *v*_*h*_ and decreases with the increase in parameters *c*, *k*.

The article "Pharmaceutical Reagent Inventory Strategy Based on Contract Shelf Life and Patient Demand" was retracted in 2023. Reasons: signs of a paper mill; suspected computer-generated content; unreliable results or conclusions; concerns about the data.

**Proposition 3 .**

The optimal output volume *p*_*t*_^*e∗*^ of the reagent manufacturer is linearly correlated with the hospital purchase volume *q*_*t*_^*e*^ under the hospital-owned inventory strategy.

**Proof**

Given a function *R*(*p*_*t*_^*e*^, *q*_*t*_^*e*^)=(*w*_*h*_+*v*_*h*_)∫_*a*_^(*q*_*t*_^*e*^ − *I*_*t*+1_^*h*^/*p*_*t*_^*e*^)^*ηg*(*η*)d*η* − *k*∫_(*q*_*t*_^*e*^ − *I*_*t*+1_^*h*^/*p*_*t*_^*e*^)_^*b*^*ηg*(*η*)d*η* − *c*, the partial derivative of this function can be obtained:

(11) $$\begin{array}{c} \frac{\partial R\left(p_{t}^{e},q_{t}^{e}\right)}{\partial p_{t}^{e}}=-\left(w_{h}+v_{h}+k\right)\frac{{\left(q_{t}^{e}-I_{t+1}^{h}\right)}^{3}}{{\left(p_{t}^{e}\right)}^{2}}g\left(\frac{q_{t}^{e}-I_{t+1}^{h}}{p_{t}^{e}}\right),\\ \frac{\partial R\left(p_{t}^{e},q_{t}^{e}\right)}{\partial q_{t}^{e}}=\left(w_{h}+v_{h}+k\right)\frac{q_{t}^{e}-I_{t+1}^{h}}{{\left(p_{t}^{e}\right)}^{2}}g\left(\frac{q_{t}^{e}-I_{t+1}^{h}}{p_{t}^{e}}\right). \end{array}$$

In turn, we have the following: (∂*p*_*t*_^*e*^/∂*q*_*t*_^*e*^)=(∂*R*(*p*_*t*_^*e*^, *q*_*t*_^*e*^)/∂*q*_*t*_^*e*^)/(∂*R*(*p*_*t*_^*e*^, *q*_*t*_^*e*^)/∂*p*_*t*_^*e*^)=(*p*_*t*_^*e*^/*q*_*t*_^*e*^ − *I*_*t*+1_^*h*^), in which (∂*p*_*t*_^*e*^/∂*q*_*t*_^*e*^) indicates that the optimal output volume of the reagent manufacturer is a reaction function about the hospital purchase volume when *q*_*t*_^*e*^ > *I*_*t*+1_^*h*^ and (∂*p*_*t*_^*e*^/∂*q*_*t*_^*e*^) > 0; i e., *p*_*t*_^*e*^ is positively correlated with *q*_*t*_^*e*^.

Further, the second-order partial derivative of (∂*p*_*t*_^*e*^/∂*q*_*t*_^*e*^) with respect to *q*_*t*_^*e*^ has (∂^2^*p*_*t*_^*e*^/∂(*q*_*t*_^*e*^)^2^)=0, showing that (∂*p*_*t*_^*e*^/∂*q*_*t*_^*e*^) is a constant greater than zero; i e., *p*_*t*_^*e*^ is linearly related to *q*_*t*_^*e*^.  Proposition 3 shows that when the reagent manufacturer's initial inventory cannot meet the hospital's purchase order, the reagent manufacturer's optimal output quantity *p*_*t*_^*e∗*^ will increase as the hospital's purchase quantity *q*_*t*_^*e*^ increases, and vice versa.

**Proposition 4 .**

Under the hospital self-operated inventory strategy, the expected return *E*(∏_*e*_^*e*^) of the hospital is a concave function of the purchase quantity *q*_*t*_^*e*^ of this in vitro diagnostic reagent, and when there is (*w*_*e*_+*v*_*e*_ − *k*)[(1 − *ηm*)*I*_*t*+1_^*h*^+*I*_*t*+1_^*e*^] − *w*_*h*_ > 0, there is a unique *q*_*t*_^*e∗*^ to maximize the expected return of the hospital, and *q*_*t*_^*e∗*^ meets the following conditions:

(12) $$\begin{array}{c} \left(w_{e}+v_{e}-k\right)\bar{F}\left(I_{t+1}+\eta m\left(q_{t}^{e}-I_{t+1}^{h}\right]\right.-w_{h}=0, \end{array}$$

where *m*=(*p*_*t*_^*e∗*^/*q*_*t*_^*e*^ − *I*_*t*+1_^*h*^) is a constant greater than 0.

The article "Pharmaceutical Reagent Inventory Strategy Based on Contract Shelf Life and Patient Demand" was retracted in 2023. Reasons: signs of a paper mill; suspected computer-generated content; unreliable results or conclusions; concerns about the data.

**Proof**

*m* is substituted into equation (7) to get (*w*_*h*_+*v*_*h*_)∫_*a*_^(1/*m*)^*ηg*(*η*)d*η*=*k*∫_(1/*m*)_^*b*^*ηg*(*η*)d*η*+*c*., and then, *m*(*q*_*t*_^*e*^ − *I*_*t*+1_^*h*^)=*p*_*t*_^*e∗*^ is substituted into equation (6) to get the hospital's income expressed as∏_*e*_^*e*^=*w*_*e*_min[*ε*, *I*_*t*+1_^*e*^+min(*q*_*t*_^*e*^, *I*_*t*+1_^*h*^+*ηm*(*q*_*t*_^*e*^ − *I*_*t*+1_^*h*^))] − *w*_*h*_min(*q*_*t*_^*e*^, *I*_*t*+1_^*h*^+*ηm*(*q*_*t*_^*e*^ − *I*_*t*+1_^*h*^)) − *v*_*e*_[*ε* − *I*_*t*+1_^*e*^ − min(*q*_*t*_^*e*^, *I*_*t*+1_^*h*^+*ηm*(*q*_*t*_^*e*^ − *I*_*t*+1_^*h*^))]^+^ − *k*[min(*q*_*t*_^*e*^, *I*_*t*+1_^*h*^+*ηm*(*q*_*t*_^*e*^ − *I*_*t*+1_^*h*^))+*I*_*t*+1_^*e*^ − *ε*]^+^. Then, the expected benefit of the hospital is further obtained as follows:

(13) $$\begin{array}{c} E\left(\prod_{e}^{e}\right)=\left(w_{e}+v_{e}-k\right)\left[\int_{a}^{\left(1/m\right)}\int_{I_{t+1}^{h}+I_{t+1}^{e}+\eta m\left(q_{t}^{e}-I_{t+1}^{h}\right)}^{+\infty }\left(I_{t+1}+\eta m\left(q_{t}^{e}-I_{t+1}^{h}\right)-x\right)f\left(x\right)\text{d}xg\left(\eta \right)\text{d}\eta +\int_{\left(1/m\right)}^{b}\int_{I_{t+1}^{e}+q_{t}^{e}}^{+\infty }\left(q_{t}^{e}+I_{t+1}^{e}-x\right)f\left(x\right)\text{d}xg\left(\eta \right)\text{d}\eta \right]\\ +\left(w_{e}-k\right)\mu_{\varepsilon }-w_{h}\left[\int_{a}^{\left(1/m\right)}\left(I_{t+1}^{h}+\eta m\left(q_{t}^{e}-I_{t+1}^{h}\right)\right)g\left(\eta \right)\text{d}\eta +\int_{\frac{1}{m}}^{b}q_{t}^{e}g\left(\eta \right)\text{d}\eta \right]. \end{array}$$

The first-order and second-order partial derivatives of the above equation with respect to *q*_*t*_^*e*^ can be obtained, respectively, as follows:

(14) $$\begin{array}{c} \frac{\partial E\left(\prod_{e}^{e}\right)}{\partial q_{t}^{e}}=\left(w_{e}+v_{e}-k\right)\bar{F}\left(I_{t+1}+\eta m\left(q_{t}^{e}-I_{t+1}^{h}\right)\right)\left[\int_{a}^{\left(1/m\right)}m\eta g\left(\eta \right)\text{d}\eta +\int_{a}^{\left(1/m\right)}g\left(\eta \right)\text{d}\eta \right]-w_{e}\left[\int_{a}^{\left(1/m\right)}m\eta g\left(\eta \right)\text{d}\eta +\int_{a}^{\left(1/m\right)}g\left(\eta \right)\text{d}\eta \right],\\ \frac{\partial^{2}E\left(\prod_{e}^{e}\right)}{\partial {\left(q_{t}^{e}\right)}^{2}}=-m\eta \left(w_{e}+v_{e}-k\right)f\left(I_{t+1}+m\eta \left(q_{t}^{e}-I_{t+1}^{h}\right)\right)\left[\int_{a}^{\left(1/m\right)}m\eta g\left(\eta \right)\text{d}\eta +\int_{a}^{\left(1/m\right)}g\left(\eta \right)\text{d}\eta \right]<0. \end{array}$$

It can be seen that the expected revenue function of the hospital is a convex function about the purchase amount of this reagent, and (∂*E*(∏_*e*_^*e*^)/∂*q*_*t*_^*e*^) is monotonically decreasing with respect to *q*_*t*_^*e*^ in the interval (0, +*∞*), and because $\underset{q_{t}^{e}⟶\infty }{\lim}\left(\partial E\left(\prod_{e}^{e}\right)/\partial q_{t}^{e}\right)=-w_{e}\left[\int_{a}^{\left(1/m\right)}m\eta g\left(\eta \right)\text{d}\eta +\int_{a}^{\left(1/m\right)}g\left(\eta \right)\text{d}\eta \right]<0$, when $\underset{q_{t}^{e}⟶0}{\lim}\left(\partial E\left(\prod_{e}^{e}\right)/\partial q_{t}^{e}\right)>0$, that is, when the condition (*w*_*e*_+*v*_*e*_ − *k*)[(1 − *ηm*)*I*_*t*+1_^*h*^+*I*_*t*+1_^*e*^] − *w*_*h*_ > 0 is satisfied, there is one and only one value *q*_*t*_^*e∗*^ in the interval (0, +*∞*) that satisfies $\left[\left(w_{e}+v_{e}-k\right)\bar{F}\left(I_{t+1}+\eta m\left(q_{t}^{e}-I_{t+1}^{h}\right)\right)-w_{h}\right]\left[\int_{a}^{\left(1/m\right)}m\eta g\left(\eta \right)\text{d}\eta +\int_{a}^{\left(1/m\right)}g\left(\eta \right)\text{d}\eta \right]=0$, and it is easy to know ∫_*a*_^(1/*m*)^*mηg*(*η*)d*η*+∫_*a*_^(1/*m*)^*g*(*η*)d*η* ≠ 0 from the assumptions, so *q*_*t*_^*e∗*^ satisfies $\left(w_{e}+v_{e}-k\right)\bar{F}\left(I_{t+1}+\eta m\left(q_{t}^{e}-I_{t+1}^{h}\right)\right)-w_{h}=0$.  Proposition 4 shows that in the case of a hospital establishing its own warehouse, there exists an optimal purchase quantity *q*_*t*_^*e∗*^ for the hospital when the parameters satisfy certain conditions, and *q*_*t*_^*e∗*^ increases with the sale price *w*_*e*_ and the out-of-stock cost *v*_*e*_ and decreases with the increase in the wholesale price *w*_*h*_ and the end-of-life cost *k* of the reagent manufacturer. At the same time, it can be seen from Proposition 2 to Proposition 4 that since *p*_*t*_^*e∗*^ and *q*_*t*_^*e∗*^ are linearly related, the system optimal decision (*p*_*t*_^*e∗*^, *q*_*t*_^*e∗*^) of the in vitro diagnostic reagent supply chain can be obtained by establishing the equation system through simultaneous equations (8) and (12). By adjusting the corresponding parameters to change the production decisions of reagent manufacturers and procurement decisions of hospitals, the supply chain can optimize the inventory and maximize the revenue of participating members of the supply chain.

The article "Pharmaceutical Reagent Inventory Strategy Based on Contract Shelf Life and Patient Demand" was retracted in 2023. Reasons: signs of a paper mill; suspected computer-generated content; unreliable results or conclusions; concerns about the data.

### 3.3. Reagent Distributor Collaborative Inventory Strategy

In this scenario, the hospital cooperates with the local distributor of the reagent manufacturer, and the hospital does not need to set up its own warehouse, but orders from the reagent manufacturer by sharing the information of patient demand and dispatches the reagent to the hospital directly from the distributor's warehouse on time, and the distributor bears the corresponding inventory management cost *τ* and is less likely to run out of stock due to the just-in-time system. The reagent manufacturer decides the output volume according to the patient consumption demand and the distributor's inventory status, and the hospital pays the corresponding unit management cost *γ* to the distributor according to the actual consumption. At this point, the hospital's revenue is expressed as follows:

(15) $$\begin{array}{c} \prod_{e}^{d}=\left(w_{e}-w_{h}-\gamma \right)\min\left(\varepsilon ,I_{t+1}+\eta p_{t}^{d}\right). \end{array}$$

The revenue of reagent manufacturers is expressed as follows:

(16) $$\begin{array}{c} \prod_{\text{h}}^{d}=w_{h}\min\left(\varepsilon ,I_{t+1}+\eta p_{t}^{d}\right)-k{\left(I_{t+1}+\eta p_{t}^{e}-\varepsilon \right)}^{+}-v_{e}{\left(\varepsilon -I_{t+1}-\eta p_{t}^{d}\right)}^{+}-cp_{t}^{d}. \end{array}$$

To simplify the model, without considering the sales of distributors and considering only their warehousing role, the distributor revenue is as follows:

(17) $$\begin{array}{c} \prod_{d}^{d}=\left(\gamma -\tau \right)\min\left(\varepsilon ,I_{t+1}+\eta p_{t}^{d}\right). \end{array}$$

Then, the total revenue of the in vitro diagnostic reagent supply chain is as follows:

(18) $$\begin{array}{c} \prod^{d}=\prod_{e}^{d}+\prod_{h}^{d}+\prod_{d}^{d}. \end{array}$$

**Proposition 5 .**

When the reagent distributor cooperates with the hospital to manage the inventory, the expected return function *E*(∏_*h*_^*d*^) of the reagent manufacturer is a concave function about the output *p*_*t*_^*d*^, and when ((*w*_*e*_+*v*_*e*_)*μ*_*η*_ − *c*/*w*_*e*_+*v*_*e*_+*k*) > *F*(*I*_*t*+1_)∫_*a*_^*b*^*ηg*(*η*)d*η*, there is a unique output *p*_*t*_^*d∗*^, which maximizes the expected return function, and *p*_*t*_^*d∗*^ satisfies the following conditions:

(19) $$\begin{array}{c} \left(w_{e}+v_{e}\right)\int_{a}^{b}\eta \bar{F}\left(I_{t+1}+\eta p_{t}^{d}\right)g\left(\eta \right)\text{d}\eta =k\int_{a}^{b}\eta F\left(I_{t+1}+\eta p_{t}^{d}\right)g\left(\eta \right)\text{d}\eta +c. \end{array}$$

**Proof**

According to formula (10), the expected revenue function of the reagent manufacturer is obtained as follows:

(20) $$\begin{array}{c} E\left(\prod_{h}^{d}\right)=w_{h}\left[\int_{a}^{b}\int_{0}^{I_{t+1}+\eta p_{t}^{d}}xf\left(x\right)\text{d}xg\left(\eta \right)\text{d}\eta +\int_{a}^{b}\int_{I_{t+1}+\eta p_{t}^{d}}^{+\infty }\left(I_{t+1}+q_{t}^{d}\right)f\left(x\right)\text{d}xg\left(\eta \right)\text{d}\eta \right]\\ -k\int_{a}^{b}\int_{0}^{I_{t+1}+\eta p_{t}^{d}}\left(I_{t+1}+q_{t}^{d}-x\right)f\left(x\right)\text{d}xg\left(\eta \right)\text{d}\eta -v_{e}\int_{a}^{b}\int_{I_{t+1}+\eta p_{t}^{d}}^{+\infty }\left(x-I_{t+1}-q_{t}^{d}\right)f\left(x\right)\text{d}xg\left(\eta \right)\text{d}\eta -cp_{t}^{d}. \end{array}$$

The first and second partial derivatives of *p*_*t*_^*d*^ are as follows:

(21) $$\begin{array}{c} \frac{\partial E\left(\prod_{h}^{d}\right)}{\partial p_{t}^{c}}=\left(w_{e}+v_{e}\right)\int_{a}^{b}\eta \bar{F}\left(I_{t+1}+\eta p_{t}^{d}\right)g\left(\eta \right)\text{d}\eta -k\int_{a}^{b}\eta F\left(I_{t+1}+\eta p_{t}^{d}\right)g\left(\eta \right)\text{d}\eta -c,\\ \frac{\partial^{2}E\left(\prod_{h}^{d}\right)}{\partial {\left(p_{t}^{c}\right)}^{2}}=-\left(w_{e}+v_{e}+k\right)\int_{a}^{b}\eta f\left(I_{t+1}+\eta p_{t}^{d}\right)g\left(\eta \right)\text{d}\eta <0. \end{array}$$

It can be seen that the expected return function *E*(∏_*h*_^*d*^) is a concave function about the supplier's output *p*_*t*_^*d*^, and (∂*E*(∏_*h*_^*d*^)/∂*p*_*t*_^*c*^) is monotonically decreasing with respect to *p*_*t*_^*d*^ in the interval (0, +*∞*), and because $\underset{p_{t}^{d}⟶0}{\lim}\left(\partial E\left(\prod_{h}^{d}\right)/\partial p_{t}^{c}\right)=\left(w_{e}+v_{e}\right)\mu_{\eta }-\left(w_{e}+v_{e}+k\right)F\left(I_{t+1}\right)\int_{a}^{b}\eta g\left(\eta \right)\text{d}\eta -c$*m*, $\underset{p_{t}^{d}⟶+\infty }{\lim}\left(\partial E\left(\prod_{h}^{d}\right)/\partial p_{t}^{c}\right)=-k\mu_{\eta }-c<0$, when $\underset{p_{t}^{d}⟶0}{\lim}\left(\partial E\left(\prod_{h}^{d}\right)/\partial p_{t}^{c}\right)>0$, that is, ((*w*_*e*_+*v*_*e*_)*μ*_*η*_ − *c*/*w*_*e*_+*v*_*e*_+*k*) > *F*(*I*_*t*+1_)∫_*a*_^*b*^*ηg*(*η*)d*η*, there is only one optimal solution *p*_*t*_^*d∗*^, which satisfies the condition: $\left(w_{e}+v_{e}\right)\int_{a}^{b}\eta \bar{F}\left(I_{t+1}+\eta p_{t}^{d}\right)g\left(\eta \right)\text{d}\eta =k\int_{a}^{b}\eta F\left(I_{t+1}+\eta p_{t}^{d}\right)g\left(\eta \right)\text{d}\eta +c$.

The article "Pharmaceutical Reagent Inventory Strategy Based on Contract Shelf Life and Patient Demand" was retracted in 2023. Reasons: signs of a paper mill; suspected computer-generated content; unreliable results or conclusions; concerns about the data.

Proposition 5 shows that in the case of collaborative inventory management by reagent distributors, when the parameters meet certain conditions reagent manufacturers have optimal output *p*_*t*_^*d∗*^ and the optimal production decision is influenced by parameters *w*_*h*_, *v*_*h*_, *c*, and *k*. By adjusting the corresponding parameters to achieve collaborative inventory control between hospitals and distributors to reduce out-of-stock loss penalties to meet patient consumption demand, the Pareto improvement of the in vitro diagnostic reagent supply chain system is realized.

## 4. Numerical Analyses

In this subsection, to verify the above mathematical model and propositional inferences, and to visually compare the effects of random output of reagent manufacturers, out-of-stock costs, and patient consumption demand on the production and purchasing decisions of participating members of the in vitro diagnostic reagent supply chain under different inventory strategies, a certain type of in vitro reagent product is selected, numerically solved using MATLAB software, and graphically analyzed using Origin software. Assuming that the random output probability *η* of reagent manufacturers obeys the uniform distribution *U*(*a*, *b*) and the consumption demand *ε* of hospital patients obeys the normal distribution *N*(*μ*_*ε*_, *σ*_*ε*_^2^), the values of other parameters are assigned as follows: *w*_*e*_=120, *w*_*h*_=100, *I*_*t*+1_^*h*^=80, *I*_*t*+1_^*e*^=20, *v*_*e*_=80, *v*_*h*_=45, *k*=120, *c*=80, *a*=0.9, *b*=1, *μ*_*ε*_=200, and *σ*_*ε*_=20, which is used as the benchmark to adjust the value range of different parameters. The effects of reagent manufacturers' random output, shortage cost, and patient consumption demand on the overall expected return and inventory of in vitro diagnostic reagent supply chain under the three strategies are discussed.

### 4.1. Influence of Reagent Manufacturer's Random Output

Let the random output probability *η* of reagent manufacturers take random values on the interval of (0, +*∞*), and other parameters are kept constant to obtain the effect of random output probability *η* on the expected profit and inventory of in vitro diagnostic reagent supply chain, as shown in Table 1 and Figure 2. From the table below, it can be seen that the overall expected return of the supply chain under the three inventory strategies is inversely correlated with the random output probability of the reagent manufacturers, and the expected return decreases as the random output probability increases, and the expected return of the supply chain under the centralized inventory decision always remains the highest, and in comparison, the overall return level under the collaborative distributor inventory strategy is the lowest, indicating that the random output probability of the hospital has a more significant effect on the inventory of the reagent distributors. From Figure 2, it can be seen that the optimal output quantity *p*_*t*_^*∗*^ of the reagent manufacturer and the optimal purchase quantity *q*_*t*_^*∗*^ of the hospital under all three inventory strategies decrease as the uncertainty of random output decreases, and the magnitude of the effect of *η* on *p*_*t*_^*∗*^ is greater than that of *q*_*t*_^*∗*^. It can also be seen that the third distributor collaborative inventory management model maintains a lower inventory quantity compared with the other two inventory management strategies, indicating that this inventory strategy is more advantageous under the influence of random output. Therefore, to maximize the overall revenue of the in vitro diagnostic reagent supply chain and optimize the inventory volume of participating supply chain members, overseas suppliers are required to strictly control the random output risk through various efforts. Table 1 is the effect of stochastic output probability on optimal decision and revenue of in vitro diagnostic reagent supply chain under three inventory strategies. Figure 2 presents the effect of random output probability on the overall inventory of in vitro diagnostic reagents supply chain.

The article "Pharmaceutical Reagent Inventory Strategy Based on Contract Shelf Life and Patient Demand" was retracted in 2023. Reasons: signs of a paper mill; suspected computer-generated content; unreliable results or conclusions; concerns about the data.

### 4.2. Influence of Hospital Out-of-Stock Punishment Cost

The trend of *v*_*e*_ on the overall revenue and inventory volume of the in vitro diagnostic reagent supply chain is shown in Figure 3 by changing the value of the hospital unit out-of-stock penalty cost *v*_*e*_. It can be seen that *v*_*e*_ has a significant effect on the supply chain expected revenue and inventory, and this is because as *v*_*e*_ increases leading to an increase in out-of-stock costs, to avoid high penalties due to out of stock, hospitals increase their purchase orders and reagent manufacturers adjust their production plans to increase production. Meanwhile, it can be seen that the expected revenue of the supply chain increases and then decreases with the penalty cost under the three strategies, which is because when *v*_*e*_ is small, i e., the situation of oversupply is easy to occur, and the supply chain system tends to reduce production and procurement in order to avoid inventory redundancy; as *v*_*e*_ increases, the procurement quantity of such reagents will increase to avoid the loss caused by stock-out; i e., the overall revenue of the supply chain increases with the improvement of patient consumption satisfaction rate. When *v*_*e*_ is maintained in a certain range, the cost of out-of-stock penalties of such reagents tends to balance with the transportation and scrap costs, and the expected revenue of the in vitro diagnostic reagent supply chain is the largest at this time, after which the expected revenue always keeps decreasing as it increases.

In addition, the expected revenue always remains highest under the centralized inventory strategy, and when *v*_*e*_ < 90, the expected revenue under the collaborative distributor inventory strategy is greater than the expected revenue under the hospital-owned inventory strategy, when increasing the unit penalty cost *v*_*e*_ is more significant to improve the overall supply chain revenue, because hospitals do not manage reagent inventory in this scenario and tend to increase purchase orders to meet patient consumption demand; when *v*_*e*_ > 90, the expected benefit under the hospital's own inventory strategy is greater than that under the distributor's collaborative inventory strategy, the reduction in the unit out-of-stock penalty cost *v*_*e*_ is more significant in enhancing the overall supply chain benefit, because the hospital bears the storage cost in this scenario, and the excessive out-of-stock cost leads to a reduction in the hospital's benefit, which also reduces the purchase order and enhances the willingness to cooperate with the distributor to manage the inventory. Figure 3 is the effect of out-of-stock penalty cost on expected revenue and inventory of in vitro diagnostic reagent supply chain.

The article "Pharmaceutical Reagent Inventory Strategy Based on Contract Shelf Life and Patient Demand" was retracted in 2023. Reasons: signs of a paper mill; suspected computer-generated content; unreliable results or conclusions; concerns about the data.

### 4.3. Influence of Patient Consumption Demand

The expected revenue of in vitro diagnostic reagent supply chain is influenced by the consumption demand of hospital patients, and according to the hypothesis condition, this secondary supply chain patient consumption demand also has uncertainty and changes the value range of *σ*_*ε*_ for sensitivity analysis to obtain Figure 4. The graph below shows that as the standard deviation of demand *σ*_*ε*_ increases, the overall expected revenue of the in vitro diagnostic reagent supply chain decreases and the supply chain inventory rises slowly. This is because the inventory and obsolescence costs of reagent manufacturers, distributors, and hospitals increase under any inventory strategy as demand uncertainty increases for this category of reagents. Meanwhile, under different standard deviation scenarios of patient consumption demand, the overall expected return of the supply chain under the centralized inventory strategy is always higher than the other two inventory strategies, and the distributor collaborative inventory strategy can maintain a lower inventory level with better expected return, indicating that the distributor collaborative inventory strategy is better than the hospital-owned inventory strategy under the increased demand uncertainty. At the same time, further analysis found that although the overall expected revenue of the supply chain decreases with the increase in the standard deviation *σ*_*ε*_ of the market demand, the expected revenue of the reagent manufacturer will increase accordingly. This is because the hospital will estimate the consumption demand of patients, and whether it stocking in warehouses or stocking up at distributors will increase purchase orders for such commodities, forcing reagent manufacturers to reduce the risk of random output to increase production. However, when the uncertainty of patient consumption demand exceeds a certain threshold, it will prompt hospitals to seek to cooperate with other reagent manufacturers or purchase alternative products. Figure 4 displays the impact of patient consumption demand standard deviation on overall expected supply chain revenue and inventory levels.

The article "Pharmaceutical Reagent Inventory Strategy Based on Contract Shelf Life and Patient Demand" was retracted in 2023. Reasons: signs of a paper mill; suspected computer-generated content; unreliable results or conclusions; concerns about the data.

## 5. Conclusions

By constructing a secondary supply chain consisting of reagent manufacturers, distributors, and hospitals, and considering the stochastic output risk of reagent manufacturers based on uncertain patient consumption demand, the theoretical idea of supplier management inventory is introduced into the in vitro diagnostic reagent supply chain, and the optimal production decision of reagent manufacturers and the optimal purchasing decision of hospitals are constructed. This study compares and analyzes the overall expected revenue, production, and procurement of the supply chain under the three inventory management strategies, studies the overall inventory optimization of the in vitro diagnostic reagent supply chain, and makes a numerical analysis with an example to demonstrate the impact of reagent manufacturers' random output risk, hospital out-of-stock penalty cost, and patients' consumption demand on the inventory optimization strategy of the in vitro diagnostic reagent supply chain.

The main conclusions are as follows: (1) the expected revenue of the in vitro diagnostic reagent supply chain under the centralized inventory strategy is a joint concave function of the production volume of reagent manufacturers and hospital purchasing volume; there is and exists a unique optimal production volume to maximize the expected revenue of reagent manufacturers and hospitals under the hospital-owned inventory strategy; when certain conditions are satisfied, there is also an optimal production volume to maximize the expected revenue of the in vitro diagnostic reagent supply chain as a whole under the collaborative inventory management strategy of distributors. (2) In comparison, with the increase in random output probability of reagent manufacturers and uncertainty of patient consumption demand, the strategy of collaborative inventory management by distributors is always better than the strategy of managing inventory by hospitals' own warehouses, which can achieve higher expected revenue and better inventory quantity, but when hospitals' out-of-stock costs are too high beyond a certain threshold, hospitals will tend to adopt the strategy of self-operated inventory. The insight is that when hospitals optimize inventory on their own or in cooperation with supply chain members, they need to take into account the random output risk of vendors to avoid supply disruptions and meet the uncertain demand of patient consumption.

The article "Pharmaceutical Reagent Inventory Strategy Based on Contract Shelf Life and Patient Demand" was retracted in 2023. Reasons: signs of a paper mill; suspected computer-generated content; unreliable results or conclusions; concerns about the data.

## Figures and Tables

**Figure 1:** In vitro diagnostic reagent supply chain procurement, production, and inventory analysis framework.

**Figure 2:** Effect of random output probability on the overall inventory of in vitro diagnostic reagent supply chain.

**Figure 3:** Effect of out-of-stock penalty cost *v*_*e*_ on expected revenue and inventory of in vitro diagnostic reagent supply chain.

**Figure 4:** Impact of patient consumption demand standard deviation *σ*_*ε*_ on overall expected supply chain revenue and inventory levels.

**Table 1:** Effect of stochastic output probability on optimal decision and revenue of in vitro diagnostic reagent supply chain under three inventory strategies.

*σ*_*ε*_	*p*_*t*_^*c*^	*q*_*t*_^*c*^	*p*_*t*_^*e*^	*q*_*t*_^*e*^	*I*_*t*+1_=*p*_*t*_^*d*^	*E*(∏^*c*^)	*E*(∏^*e*^)	*E*(∏^*d*^)
(0,1)	445.5	193.5	463.5	180	426	−2298.63	−2594.01	−2466.47
(0.1,1)	423	192	445.5	180	405	−1521.18	−1953.72	−1781.57
(0.2,1)	403.5	192	429	178.5	385.5	−852.555	−1128.96	−935.595
(0.3,1)	385.5	190.5	397.5	178.5	361.5	−17.67	−175.23	−130.41
(0.4,1)	348	190.5	364.5	175.5	340.5	722.085	665.55	684.315
(0.5,1)	324	187.5	328.5	175.5	319.5	1461.84	1358.64	1385.535
(0.6,1)	289.5	187.5	294	175.5	283.5	2201.595	2058.93	2126.295
(0.7,1)	261	186	253.5	172.5	256.5	2941.35	2780.16	2840.46
(0.8,1)	235.5	186	222	172.5	238.5	3681.12	3484.545	3555.6
(0.9,1)	204	183	190.5	169.5	214.5	4314.345	4115.88	4151.7
(0.95,1)	202.5	183	189	169.5	214.5	4325.415	4110.87	4177.05
(0.99,1)	201	183	187.5	169.5	213	4338.225	4125.225	4190.295

## Data Availability

The simulation experiment data used to support the findings of this study are available from the corresponding author upon request.
